# Development of a Robotic Catheter Manipulation System Based on BP Neural Network PID Controller

**DOI:** 10.1155/2020/8870106

**Published:** 2020-12-23

**Authors:** Xu Ma, Jinpeng Zhou, Xu Zhang, Qi Zhou

**Affiliations:** ^1^Tianjin Key Laboratory for Control Theory & Applications in Complicated Industry Systems, College of Electrical and Electronic Engineering, Tianjin University of Technology, Tianjin, China 300384; ^2^Tianjin Key Laboratory of High Speed Cutting and Precision Machining, School of Mechanical Engineering, Tianjin University of Technology and Education, Tianjin, China 300222

## Abstract

In the process of artificial interventional therapy, the operation of artificial catheter is not accurate, which will bring strong radiation damage to surgeons. The purpose of this study is to develop a catheter operating system of surgical robot to assist doctors in remote operation and avoid the influence of radiation. BP neural network plays an important role in the flexibility and rapidity of control. According to the actual output of the system, the control parameters of the controller are constantly adjusted to achieve better output effect. This paper introduces the practical application of BP neural network PID controller in the remote operation of the system and compares with the traditional PID controller. The results show that the new control algorithm is feasible and effective. The results show that the synchronization performance of BP neural network PID controller is better than that of traditional PID controller.

## 1. Introduction

Vascular interventional surgery in medicine, whether from the diagnosis or the actual operation, has been welcomed by the society. However, as a new way of operation, it needs surgeons with high skill to intubate in vivo. In addition, the interventional operation is carried out in the patient's body, and the specific process cannot be directly observed by the doctor. During the operation, any incorrect operation may cause damage to the patient. According to the data survey, a surgeon with rich clinical experience can achieve an operation accuracy of about 2 mm in the interventional operation. However, the contact force between the blood vessels in the patient's body and the surgical catheter cannot be perceived by the doctor [1]. In addition, X-ray camera is needed for angiography during the operation, and long-term radiation will cause harm to patients. Although doctors wear protective clothing, it is difficult to protect their hands and faces from X-ray radiation. In order to solve these problems effectively, we need better medical equipment to assist doctors [2]. The robot system has the advantages of high control accuracy and remote control. Therefore, in this paper, according to the needs of interventional surgery, combined with the robot system, the master-slave operating system of interventional surgery robot which can assist doctors in interventional surgery is designed [3].

There are a large number of products and research reports in the field of surgical robots [4]. One of the most popular commercial products is the Sensei robotic catheter system designed and developed by Hansen, which is mainly to help doctors push the catheter. Compared with the manual push, the Sensei robot catheter system can make the push process more stable and rapid, and the operation accuracy is higher. The remote control method can reduce the original radiation impact of doctors. Another commercial product is amigo, which is mainly designed to solve the problem that the sheath of the surgical catheter has multiple degrees of freedom and the force detection at the end of the catheter is difficult. The robotic catheter system has an additional mechanical sheath to guide the surgical catheter [5]. The pushing process of the surgical catheter is controlled by the console at the host end. In 2010, Magnetecs Company got the design inspiration from the treatment of atrial fibrillation and designed a system that can use magnetic field to guide, control, and image the surgical catheter in British. The system consists of four permanent magnets placed around the table, and the top of the designed surgical catheter is equipped with magnets. The catheter moves in the magnetic field under the control of the console at the main end. With the popularity of surgical robots, stereotactic companies have also developed a magnetic navigation system: Stereotactic Niobe. The system can generate controllable magnetic field by two permanent magnets on both sides of the operating table, reduce the number of permanent magnets, and make the navigation of magnetic guide wire more convenient and accurate in percutaneous coronary intervention (PCI). In other universities, Ma and others developed a catheter navigation system that can be operated remotely [6]. The system allows the main end operator to use the real surgical catheter instead of the handle to control the movement of the surgical catheter in the patient's body. This progress can make the doctor's original surgical experience applied to the actual operation. However, the system is lack of force feedback, which operational safety cannot be guaranteed. In order to simulate the use of doctors' hands, Bao et al. proposed a special linear step structure in Nagoya University. Based on the above products and academic research, the main problem lies in the security of system operation [8]. During the operation, it is an important step to monitor the force information of the catheter inserted into the blood vessel to ensure the safety of the operation. However, in these systems, there is a lack of effective measurement of conduit stress [8].

In this paper, according to the operation needs of vascular interventional surgery, a new robot operation system of surgical catheter is designed and constructed. Compared with the abovementioned surgical robot system, the system is also divided into two parts: one is the main end of the robot catheter manipulating system, as shown in Figure 1(a), which is mainly used to collect the axial displacement and radial rotation movement of the operator, consisting of pressure sensor, torque sensor, stepping motor, and controller. The other is the slave end of the robot catheter manipulating system, which is mainly used for the insertion and twisting operation of the conduit is shown in Figure 1(b). In addition, aiming at the safety of force detection, the research team designed a new force feedback detection device, which can detect the change of contact force between the catheter and the vessel wall during the insertion of the surgical catheter from the end of the system [9], and timely provide force feedback to the main end of the system to ensure the safety of the operation [10].

## 2. Robotic Catheter Manipulation System

In this paper, the main mode of master-slave operation is adopted. The main end of the system is the surgeon's console, and the slave end of the system is the surgical catheter console. Setting the mobile platform of the main end doctor console and the slave end catheter console to maintain the same displacement, speed and rotation angle will make the operation more stable and convenient [11]. At the same time, the same digital signal processor (Ti, TMS320F28335) is used as the control unit of the master doctor console and the slave catheter console [12]. The main end and the slave end of the surgical robot system establish a communication network through the Internet, and the communication diagram is shown in Figure 2. The console at the main end of the system transmits the axial displacement and radial rotation motion information of the mechanical handle to the catheter console at the slave end to perform specific operation. Set the baud rate of the communication serial port between the master and slave of the system to 19200 B/s [13].

### 2.1. The Surgeon's Console

The doctor's console at the main end of the system is shown in Figure 1(a). Two independent sensors are used to measure the axial and radial movement of the mechanical handle. The switch on the left mechanical handle is used to control the two graspers on the console of the slave end conduit of the system to help realize the insertion process of the slave end conduit. The mechanical handle on the right is used to collect the specific actions of the surgeon, including the axial movement and the radial movement. The moving part of the slave end conduit console maintains the same amount of movement as the right mechanical handle of the main end console. The mechanical handle on the right side of the main end is supported by the mechanical bearing and connected with the load cell through the coupling; the pulley are fixed on the mechanical handle for the convenience of force transmission.

The measurement process of the axial movement of the mechanical handle is as follows. When the doctor pulls or pushes the right mechanical handle, the load cell measures the pull/push force. According to the thrust value, the corresponding displacement of the mobile platform is calculated, that is, the mechanical handle can follow the synchronous movement of the surgeon's hand. By adjusting the moving speed of the mobile platform, the force feedback of the system can be realized. The displacement and speed information of the system's main end console is sent to the system's slave end console, and then, the slave end catheter console and the main end doctor console are set to keep synchronous motion. When the doctor turns the mechanical handle, the mechanical encoder installed under the main end moving platform will drive the encoder, then measure the actual angle, and transmit the measured value to the slave end catheter console for synchronous movement. In this way, the implementation process of the master side operation in the slave side is realized.

### 2.2. The Surgical Catheter Console

Figure 1(b) shows the conduit console at the slave end of the system. The device is placed next to the patient. The catheter console can assist doctors to push the catheter. It has two degrees of freedom: axial displacement and radial rotation. Two clips are placed in the pushing guide, and the switch of the clips is controlled by the button on the left mechanical handle of the main end. When the surgical catheter is clamped by the grasper 1 and the jacket together, the movement of the main end doctor to the mechanical handle can be realized, and the synchronous movement of the slave end surgical catheter along the axial and radial directions can be driven [14]. When the surgical catheter is clamped by the grasper 2, the catheter maintains its position, and then, the catheter driving part at the end can move freely to prepare for the next push. The pushing action of the catheter from the end of the operation is shown in Figure 3.

In order to achieve the axial movement of the conduit, all the driving components are fixed on the mobile platform (the flat plate under the motor 1). The mobile platform is driven by a stepping motor (motor 2) to achieve axial movement. The radial movement of the conduit needs to be realized by the DC motor (motor 1), which is realized by the jacket connected by two pulleys. When the surgical catheter is fixed by the grasper 1, the surgical catheter is driven by the motor 1 to rotate.

The robot system uses the torque sensor installed at the slave end of the system to measure the actual rotation information of the catheter during the operation. The torque data will be sent to the surgeon's console at the main end, and the actual torque will be fed back to the surgeon. The specific working process is that the torque sensor is connected with the motor 1 and the pulley on a common shaft. In the process of pushing conduit, the resistance of conduit rotation can be transmitted to the torque sensor through the coupling pulley, and then, the actual resistance value can be measured by the torque sensor.

In order to measure the axial resistance of the catheter during pushing, a new force measuring mechanism is designed, which is shown in Figure 4 [15]. Use the load cell fixed on the mobile platform to measure the resistance value. The measured resistance value is sent to the main end of the system. Combined with the push/pull value of the doctor to the mechanical pusher, the system force feedback is realized.

### 2.3. Control of the System

At the slave end of the system, each motor is coupled to the coder. The speed and angle of rotation of these motors can be measured. Therefore, it is necessary to design control algorithms to improve the operation accuracy and motion performance of surgical robot system in remote operation. At the main end of the system, the mechanical handle should be able to move smoothly with the surgeon's hand. This means that the output displacement/speed of the stepper motor should be the same as or similar to the input displacement/speed of the surgeon's hand. The speed and displacement of the stepping motor can be measured by an encoder coupled to the motor 2 in Figure 1(b). Therefore, it is necessary to determine the axial and radial dynamic models of the surgical robot system and establish the relationship between the input force of the main end and the displacement output of the stepper motor. In terms of synchronous tracking performance, a PID controller based on BP neural network is adopted to improve the accuracy of axial displacement during remote operation [16].

## 3. BP Neural Network

Due to the high requirements for the positioning of surgical catheter in interventional surgery, it is difficult to accurately establish the control model of interventional surgery robot system due to the influence of nonlinear factors such as blood flow and vascular wall in human blood vessels, which has the risk of vascular damage. Based on the analysis of the related motion control algorithm, combined with the technical requirements of catheter propulsion accuracy and collision force in interventional surgery, a PID controller based on BP neural network is designed. Through MATLAB simulation, the control accuracy of the designed controller is verified.

### 3.1. Neural Network Theory

Figure 5 shows a simple artificial neuron model, the “M–P neuron” model. In this neuron model, each neuron receives input signals from other n neurons. After entering the neuron, these input signals will be weighted and then transmitted to the next step [17]. In the process of transmission, the weighted signal value is compared with the threshold set by neurons. If not, the neurons are not activated if they are not transferred down [18].

The model consists of multiple inputs *x*_*i*_, *i* = 1, 2, ⋯, *n* and a single output *y*. The expression for *y* is as follows:

(1) $$\begin{array}{c} y=f\left(\overset{n}{\underset{i=1}{\sum }}w_{ji}x_{i}-\theta_{j}\right), \end{array}$$

where *θ*_*j*_ is the threshold, *w*_*ji*_ is the connection weight (*w*_*ji*_ is positive in the excited state; *w*_*ji*_ is negative in the suppressed state), *n* is the number of input signals, and *f*() is the activation function.

### 3.2. The Definition and Characteristics of BP Neural Network

BP neural network is a kind of feedforward multilayer network, including input layer, implicit layer, and output layer [19]. The neurons in the same layer of BP neural network are not connected with each other, and the neurons in the upper and lower layers are connected [20].

Figure 6 shows the network structure of simple BP neural network. It consists of input layer, hidden layer, and output layer. The connection weights of the *j*-th neuron in the input layer and the *i*-th neuron in the hidden layer are *w*_*ij*_, and the weight between the *i*-th neuron in the hidden layer and the *l*-th neuron in the output layer is *w*_*li*_. The input value of the *i*-th neuron in the hidden layer is net_*i*_^(2)^ = ∑_*j*=1_^*m*^*w*_*ij*_^(2)^*ο*_*j*_^(1)^. The input value of the *l*-th neuron in the output layer is net_*l*_^(3)^ = ∑_*i*=1_^*q*^*w*_*li*_^(3)^*ο*_*i*_^(2)^. Finally, the output value of the whole neural network is obtained after the weighted sum calculation [21].

BP neural network has the following characteristics in information processing [22]:

1. Distributed storage. The weights of neurons in each layer of BP neural network represent the information of the whole network. Therefore, all information is distributed and stored through the network, and its fault tolerance is relatively high
2. Parallel processing of information. All neurons in the BP neural network are relatively independent. The neurons in the same layer are simultaneously processed by signal processing, and the whole network has better real-time performance
3. Adapt ability. The connection strength of the BP neural network increases with use, which increases the sensitivity of each neuron

### 3.3. Self-Learning of BP Neural Network

The BP neural algorithm proposed in this paper is based on gradient descent that is to adjust the parameters in the direction of negative gradient of the expected target. The details are as follows: three layer network structures, such as *m* neurons in the input layer, *q* neurons in the hidden layer, and *r* neurons in the output layer.

#### 3.3.1. Information Forward Propagation

The output of the *j*-th node of the input layer is as follows:

(2) $$\begin{array}{c} {{ο}_{j}}^{\left(1\right)}=x\left(j\right),j=1,2,\cdots ,m. \end{array}$$

Then, the output of the input layer is weighed and summed; it is the input of the *i*-th neuron of the hidden layer.

(3) $$\begin{array}{c} {{\text{net}}_{i}}^{\left(2\right)}=\overset{m}{\underset{j=1}{\sum }}{w_{ij}}^{\left(2\right)}{{ο}_{j}}^{\left(1\right)},i=1,2,\cdots ,q. \end{array}$$

After activating the function operation, the hidden layer output is as follows:

(4) $$\begin{array}{c} {{ο}_{i}}^{\left(2\right)}=f\left({{\text{net}}_{i}}^{\left(2\right)}\right),i=1,2,\cdots ,q. \end{array}$$

The superscripts (1), (2), and (3) represent the input layer, the hidden layer, and the output layer, respectively. *W*_*ij*_^(2)^ is the weight of the input layer to the hidden layer, and *f*() is the hidden layer activation function.

The output of the hidden layer is the input of the *l*-th neuron of the output layer after the weight summation calculation.

(5) $$\begin{array}{c} {{\text{net}}_{l}}^{\left(3\right)}=\overset{q}{\underset{i=1}{\sum }}{w_{li}}^{\left(3\right)}{o_{i}}^{\left(2\right)},l=1,2,\cdots ,r. \end{array}$$

The output of the output layer is as follows:

(6) $$\begin{array}{c} y_{l}={o_{l}}^{\left(3\right)}=g\left({{\text{net}}_{l}}^{\left(3\right)}\right),l=1,2,\cdots ,r, \end{array}$$

where *w*_*li*_^(3)^ is the weight of the hidden layer to the output layer; *g* is the output layer excitation function.

#### 3.3.2. Error Backpropagation [23]

If there is a large error between the actual output value and the initial set value in BP neural network, the closed-loop regulation will feed the error back to the initial end of the system for regulation. At the same time of system output, the output value of the system gradually approaches to the initial set value by continuously adjusting the weight of each network in the system. The adjustment block diagram is shown in Figure 7.

In this paper, the mean square error of BP network is selected as the standard function of evaluation, and the weight of each layer network in the system is adjusted. The mean square error is defined as follows:

(7) $$\begin{array}{c} E=\frac{1}{r}\overset{r}{\underset{l=1}{\sum }}{e_{l}}^{2}=\frac{1}{r}\overset{r}{\underset{l=1}{\sum }}{\left({y_{l}}^{*}-y_{l}\right)}^{2}, \end{array}$$

where *y*_*l*_^∗^ is the given value of the *l*-th output node; *y*_*l*_ is the actual value of the *l*-th output node.

Let *k* be the number of iterations; then, the implicit layer to output layer weight correction formula is as follows:

(8) $$\begin{array}{c} {w_{li}}^{\left(3\right)}\left(k+1\right)={w_{li}}^{\left(3\right)}\left(k\right)+\Delta {w_{li}}^{\left(3\right)}={w_{li}}^{\left(3\right)}\left(k\right)-\eta \frac{\partial E\left(k\right)}{\partial {w_{li}}^{\left(3\right)}\left(k\right)}, \end{array}$$

where *η* is a constant, indicating the learning rate, *l* = 1, 2, ⋯, *r*, *i* = 1, 2, ⋯, *q*.

The total error surface's gradient vector replace the output value *y*_*l*_ into Equation (8). Then we can adjust the hidden layer's connection weight to the output layer. Similarly, the connection weight from input layer to hidden layer can be adjusted to gradually reduce the error of the whole system, so that the system can meet the expected requirements.

Figure 8 shows the network topology of BP neural network PID controller. The input signal of the system enters the BP neural network through the network input layer. After weighted processing, it is compared with the neuron threshold and then enters the excitation function as the output of the input layer, that is, the input of the hidden layer. After processing, the output signal of the hidden layer is obtained. After entering the output layer for processing, the final output value of the system is obtained. The actual output value is compared with the expected value, and then, the error signal is fed back from the output layer to the hidden layer twice and then transmitted back to the input layer. In the whole feedback regulation process, the connection weights of each layer of neurons are modified by the error gradient descent algorithm, so that the actual output of the input signal can be corrected after entering the neural network again, so as to achieve the purpose of self-tuning of PID control parameters and finally achieve the good response of the whole system.

The topological structure of BP neural network proposed in this paper consists of three input nodes, six implicit nodes, and three output nodes. The input signal is the motion state and system error of the motor system, and the output signal is the three parameters of PID.

#### 3.3.3. Network Information Forward Propagation Calculation

(9) $$\begin{array}{c} \text{Select three inputs as }\left\{\begin{array}{c} {{ο}_{2}}^{\left(1\right)}=e\left(k\right),\\ {{ο}_{2}}^{\left(1\right)}=e\left(k-1\right),\\ {{ο}_{3}}^{\left(1\right)}=1. \end{array}\right. \end{array}$$

The input and output of the hidden layer are as follows:

(10) $$\begin{array}{c} {{\text{net}}_{i}}^{\left(2\right)}\left(k\right)=\overset{m}{\underset{j=0}{\sum }}{w_{ij}}^{\left(2\right)}{{ο}_{j}}^{\left(1\right)}, \end{array}$$

(11) $$\begin{array}{c} {{ο}_{i}}^{\left(2\right)}\left(k\right)=f\left({{\text{net}}_{i}}^{\left(2\right)}\left(k\right)\right),i=1,2,\cdots , \end{array}$$

(12) $$\begin{array}{c} \left\{\begin{array}{c} {{ο}_{i}}^{\left(2\right)}\left(k\right)=f\left({{\text{net}}_{i}}^{\left(2\right)}\left(k\right)\right)\\ {{ο}_{6}}^{\left(2\right)}\left(k\right)=1 \end{array},\right.\;i=1,2,\cdots , \end{array}$$

where *j* denotes the number of the input layer node; *i* denotes the number of the hidden layer; superscripts (1), (2), and (3) decibels represent the input, implicit, and output layers, respectively; *w*_*ij*_^(2)^ is the input layer; *j* is the weight value of the *i*-th hidden layer's node.

The excitation function *f*(*x*) is a hyperbolic tangent function:

(13) $$\begin{array}{c} f\left(x\right)=\tanh\left(x\right)=\frac{e^{x}-e^{-x}}{e^{x}+e^{-x}}. \end{array}$$

#### 3.3.4. Network Error Backpropagation Calculation

The gradient descent algorithm is used to adjust the weight coefficient value, and the performance index function is selected as follows:

(14) $$\begin{array}{c} E=\frac{1}{2}e^{x}\left(k\right). \end{array}$$

Let the error function *E* adjust in the direction of the fastest change to reduce, that is, adjust the network connection weight coefficient according to the negative gradient direction of the error function *E*, so that the error converges gradually. There is

(15) $$\begin{array}{c} \Delta {w_{li}}^{\left(3\right)}\left(k\right)=-\eta \frac{\partial E\left(k\right)}{\partial {w_{li}}^{\left(3\right)}}. \end{array}$$

In order to speed up the error correction and reduce the probability of the system falling into the local minimum, the momentum factor is added. There is

(16) $$\begin{array}{c} \Delta {w_{li}}^{\left(3\right)}\left(k\right)=-\eta \frac{\partial E\left(k\right)}{\partial {w_{li}}^{\left(3\right)}}+\alpha \Delta {w_{li}}^{\left(3\right)}\left(k-1\right), \end{array}$$

where *η* is the learning rate and *α* is the momentum factor.

According to the gradient descent method,

(17) $$\begin{array}{c} \frac{\partial E\left(k\right)}{\partial {w_{li}}^{\left(3\right)}}=\frac{\partial E\left(k\right)}{\partial y\left(k\right)}\cdot \frac{\partial y\left(k\right)}{\partial u\left(k\right)}\cdot \frac{\partial u\left(k\right)}{\partial {{ο}_{l}}^{\left(3\right)}\left(k\right)}\cdot \frac{\partial {{ο}_{l}}^{\left(3\right)}\left(k\right)}{\partial {{\text{net}}_{l}}^{\left(3\right)}\left(k\right)}\cdot \frac{\partial {{\text{net}}_{l}}^{\left(3\right)}\left(k\right)}{\partial {w_{li}}^{\left(3\right)}}. \end{array}$$

In Equation (17), the variable *∂y*(*k*)/*∂u*(*k*) is unknown, but *u*(*k*), *y*(*k*), and the relative change amount can be obtained, so

(18) $$\begin{array}{c} \frac{\partial y\left(k\right)}{\partial u\left(k\right)}=\frac{y\left(k\right)–y\left(k-1\right)}{u\left(k\right)–u\left(\text{k}-1\right)}. \end{array}$$

Since *u*(*k*) = *u*(*k* − 1) + *ο*_1_^(3)^(*e*(*k*) − *e*(*k* − 1)) + *ο*_2_^(3)^*e*(*k*) + *ο*_3_^(3)^(*e*(*k*) − 2*e*(*k* − 1) + *e*(*k* − 2)), so

(19) $$\begin{array}{c} \left\{\begin{array}{c} \frac{\partial u\left(k\right)}{\partial {{ο}_{1}}^{\left(3\right)}\left(k\right)}=e\left(k\right)-e\left(k-1\right),\\ \frac{\partial u\left(k\right)}{\partial {{ο}_{2}}^{\left(3\right)}\left(k\right)}=e\left(k\right),\\ \frac{\partial u\left(k\right)}{\partial {{ο}_{3}}^{\left(3\right)}\left(k\right)}=e\left(k\right)-2e\left(k-1\right)+e\left(k-2\right). \end{array}\right. \end{array}$$

### 3.4. The Structure of BP Neural Network PID Controller

In order to improve the control system of traditional PID controller, other intelligent optimization algorithms are combined with traditional PID controller to achieve better control effect. Among them, BP neural network algorithm as a classic intelligent optimization algorithm has the characteristics of distributed storage, parallel processing, and adaption, which makes up for the shortcomings of traditional PID controller. Therefore, the combination of BP neural network algorithm and traditional PID control can achieve the purpose of optimizing the control effect. Through the adaptive characteristics of BP algorithm, combined with input and output samples, the BP neural network model is trained, and the connection weights in the network are constantly adjusted to make the output meet the expected requirements and reduce the system error. This combined optimization control method, especially for the servo motor control system, can effectively solve the design problems that the motor PID control parameters are difficult to adjust and the overall control of the system cannot achieve the desired effect.

Figure 9 shows the system diagram of BP neural network PID controller. It is an organic combination of traditional PID controller and BP neural network. The specific contents of each part are as follows:

#### 3.4.1. BP Neural Network Part

BP neural network is an important part of BP neural network PID system. The main function is to modify the connection weight of each layer of neural network according to the actual input and output through the self-learning characteristics of BP algorithm, so as to achieve the purpose of adjusting the output, that is to adjust the control parameters of PID controller in real time and optimize the performance of the whole control system. The output signal of input layer in BP neural network corresponds to three control parameters *K*_*p*_, *K*_*i*_, and *K*_*d*_ in traditional PID controller. The adjustment process of control parameters is shown in Figure 10.

#### 3.4.2. Traditional PID Part

BP neural network is only an abstract optimization algorithm, and the actual control of the motor still depends on the traditional PID controller. Therefore, the traditional PID part is an indispensable part of the BP neural network PID system. The specific control of the motor is still dependent on the closed-loop control of the traditional PID controller, so that the motor's speed output follows the input.

### 3.5. BP Neural Network PID Controller

Taking the axial motion of the surgical robot designed in this paper as an example, the dynamic analysis is carried out. Its axial movement is driven by Maxon EC32 motor. The motor drives the system to move back and forth from the whole clamping catheter platform at the end, so as to realize the purpose of pushing the surgical catheter. According to Newton's second law of physics, after simplifying the reference factors of the system, the dynamic model of the axial motion of the surgical robot is established as follows:

(20) $$\begin{array}{c} f\left(t\right)=m\ddot{x}\left(t\right)+c\dot{x}\left(t\right)+kx\left(t\right), \end{array}$$

where *f*(*t*) is the motor driving force, *x*(*t*) is the displacement of this motion, $\dot{x}\left(t\right)$ is the motion velocity, $\ddot{x}\left(t\right)$ is the motion acceleration, and Equation (20) illustrates the relationship of motor drive force and output displacements.

If *x*_1_(*t*) = *x*(*t*) and $x_{2}\left(t\right)=\dot{x}\left(t\right)$, then,

(21) $$\begin{array}{c} \left\{\begin{array}{c} \dot{x}\left(t\right)=AX\left(t\right)+Bu\left(t\right),\\ y\left(t\right)=CX\left(t\right), \end{array}\right. \end{array}$$

where $X\left(t\right)=\left[\begin{array}{c} x_{1}\left(t\right)\\ x_{2}\left(t\right) \end{array}\right]$, $A=\left[\begin{array}{cc} 0 & 1\\ -k/m & -c/m \end{array}\right]$, $B=\left[\begin{array}{c} 0\\ 1/m \end{array}\right]$, and $C=\left[\begin{array}{cc} 1 & 0\\ 0 & 0 \end{array}\right]$.

That *m* is the mass of the overall axial movement of the push platform, *c* is the overall damping coefficient of the push platform, and *k* is the overall elastic coefficient of the push platform. From Equation (22), it can be concluded that the transfer function of the axial movement of the push device is as follows:

(22) $$\begin{array}{c} H\left(s\right)=\frac{m}{{ms}^{2}+cs+k}. \end{array}$$

### 3.6. Simulation Analysis

Taking the axial motion of the interventional robot as an example, the step signal *y* = 1 is used to simulate the axial expected displacement of the main hand catheter during the actual operation of the doctor. Take Equation (22)as *m* = 1 kg, *c* = 0.05 N/(m/s), and *k* = 1.5 N/m. After MATLAB simulation, the simulation results shown in Figure 11 are obtained and the results are in BP for comparison control effects.

Figure 11 shows the simulation comparison between BP neural network PID control and traditional PID control. By comparing the simulation results, it can be found that the overshoot of the traditional PID control system is 22%, while that of the newly designed BP neural network PID control system is only 12%. Compared with the traditional PID control system, the adjustment time and precision of BP neural network PID control system have been greatly improved. In the actual operation process, the pushing process of the surgical catheter needs several times to push and pull the catheter to reach the designated lesion. Shortening the pushing time of the catheter is helpful to improve the efficiency of intubation and the success rate of operation.

## 4. Experiments

### 4.1. Experimental Setup

The simulation experiment is made up of the RCMS which is composed of the main terminal (surgeon console) and the slave terminal (surgical catheter console) by remote operation and connected by network communication. The operation catheter was driven by step motor and DC motor for axial and radial movement. Therefore, in the process of using, it is helpful to monitor the motion state of stepping motor and DC motor for practical application and control. The BP neural network with double input and single output structure is used as the adjusting module of the control parameters in the PID controller. The displacement error (*e*(*k*)) and the change of displacement error (*ce*(*k*)) are regarded as two inputs of the controller. The realization process of the new controller is as follows: monitoring the current output value of step motor or DC motor; calculating the movement error and error change speed through the current value; inputting the error into BP neural network; and adjusting it through self-learning characteristics. Then, the adjusted *K*_*p*_, *K*_*i*_, and *K*_*d*_ are transmitted to PID controller to adjust the output signal *u*(*t*) of the whole system.

### 4.2. Experimental Results

First of all, we use the traditional PID controller to carry out the basic remote operation experiment. Then, the new designed BP neural network PID controller is used to carry out the same remote operation experiment. The experimental results of traditional PID axial displacement are shown in Figure 12, and the error of traditional PID axial displacement is shown in Figure 13.  Figure 14 shows that BP neural network PID controller obtains smooth response without overshoot, and its axial displacement error curve is shown in Figure 15.

The steady-state error of traditional PID controller is large, and the synchronous tracking performance is far inferior to that of BP neural network PID controller. However, although the BP neural network PID controller has good effect, it also has some errors. These errors are due to time delays in remote operations. This is also a key technical issue to be considered in future research.

Of course, for the axial motion of the system, we only use a simple physical method to establish the system dynamics model, without considering the higher requirements of the system in different working environments or other nonlinear factors. For a system with two degrees of freedom (radial rotation and axial displacement), when the displacement velocity or rotation direction changes, the system operation will be affected by nonlinear factors. Therefore, for the system, the nonlinear dynamic factors should be added to the known model in order to enhance the anti-interference ability of the control system and achieve better control effect.

## 5. Conclusions and Future Work

The system is based on the catheter robot operating system (RCMS), including a mechanical system with high precision and remote operation to assist surgeons in vascular intervention. The system takes digital signal processor (DSP) as the control unit, and has high measurement accuracy and processing speed in the main terminal console and the slave terminal console. Load cell and torque sensor are used to obtain the motion information of force and rotation angle. A new controller, BP neural network PID controller, is designed, which can improve the axial and rotary motion accuracy of the system in remote operation. Simulation results show that the proposed BP neural network PID controller has good dynamic response quality. When BP neural network PID controller is used for remote control, the synchronous tracking error of axial displacement is less than 1.5 mm. Although there are some errors in radial rotation and axial displacement due to time delay, the system can also meet the actual requirements of minimally invasive surgery. In conclusion, BP neural network PID control algorithm can improve the control performance of the system.

In the future research work, we will add the dynamic model of radial rotation in the operation system of surgical catheter robot, and increase the nonlinear influence factors. Combined with the established dynamic model of axial displacement, we will improve the control accuracy and anti-interference ability of the system in remote control [24]. In addition, more advanced sensors are used to measure the force (contact force and friction force) and displacement information in the system. And for the perfect system, real animal experiments were carried out to verify the reliability and safety of the system and ensure the feasibility of operation.

## Figures and Tables

**Figure 1:** The robotic catheter manipulating system.

**Figure 2:** The communication diagram.

**Figure 3:** Pushing action.

**Figure 4:** Axial force measurement mechanism.

**Figure 5:** The model of artificial neuron.

**Figure 6:** The formation of BP neural network.

**Figure 7:** The adjustment process of BP neural network.

**Figure 8:** The diagram of BP neural network structure.

**Figure 9:** The control system of BP neural network PID controller.

**Figure 10:** Intelligent adjustment output of parameters *K*_*p*_, *K*_*i*_, and *K*_*d*_.

**Figure 11:** Simulation results.

**Figure 12:** Axial displacement of PID controller.

**Figure 13:** Axial displacement error of PID controller.

**Figure 14:** Axial displacement of BP neural network PID controller.

**Figure 15:** Axial displacement error of BP neural network PID controller.

## Data Availability

The article data used to support the findings of this study are available from the submitting author upon request.
